The article "Stability Analysis and Construction Parameter Optimization of Tunnels in the Fractured Zone of Faults" was retracted in 2023. Reasons: signs of a paper mill; suspected computer-generated content; unreliable results or conclusions; concerns about the data.

# Stability Analysis and Construction Parameter Optimization of Tunnels in the Fractured Zone of Faults

**DOI:** 10.1155/2022/2211499

**Published:** 2022-08-31

**Authors:** Banma Huang, Haibo Chen, Chenglong Duan, Wenhu Li

**Affiliations:** ^1^Qinghai Traffic Engineering Technical Service Center, Xining, Qinghai 810001, China; ^2^China-Road Transportation Verification and Inspection Hi-Tech Co., Ltd., Beijing 100088, China

## Abstract

In order to improve the construction method of highway tunnel fault, improve the excavation level, improve the construction efficiency, reduce the project cost, and shorten the construction period, so as to find a specific road, this paper puts forward the research method of tunnel stability analysis and construction parameter optimization in the fault fracture zone. First, this paper analyzes the specific geographical and geological environment of the construction site. Second, this paper compares and analyzes the effects of the drilling and blasting method and full-face tunnel boring machine (TBM) in construction and further analyzes the surrounding rock deformation, over excavation, and under excavation, as well as the range of loose circles when the surrounding rock is stable. Then, this paper discusses the minimum smooth blasting parameters under these conditions. Finally, the actual blasting effect of tunnel construction is tested and the optimization algorithm model of tunnel fault drilling and blasting parameters is established. The results show that the proposed optimization model of drilling and blasting construction parameters for highway tunnel faults based on the Support Vector Regression (SVR) algorithm combined with a genetic algorithm (GA) has a short calculation time and high parameter optimization accuracy. It is very feasible to optimize the construction parameters of the fault drilling and blasting method, which can greatly improve the construction efficiency, carry out the detailed simulation, reduce the cost, and increase safety. In summary, it has a certain reference significance for the optimization of highway tunnel construction and future research by drilling and blasting method under complex geological conditions in my country.

## 1. Introduction

With the development of new infrastructure in China, new construction technology and its auxiliary means have been paid more and more attention by the engineering community. Due to the geographical and geological conditions of our country, the drilling and blasting method has become one of the main methods of tunnel construction in our country. The blasting effect of the drilling and blasting method will have a significant impact on the construction progress of the entire expressway tunnel and is of great significance to the surrounding rock and later maintenance of the tunnel [1, 2].

The article "Stability Analysis and Construction Parameter Optimization of Tunnels in the Fractured Zone of Faults" was retracted in 2023. Reasons: signs of a paper mill; suspected computer-generated content; unreliable results or conclusions; concerns about the data.

There are generally two tunneling methods for expressway tunnel faults, namely, the drilling and blasting method [3] and the tunnel boring machine (TBM) method [4]. The drilling and blasting method involves the use of rock mass drilling, laying explosives, and fixed-point blasting to excavate the tunnel. Its construction effect will be affected by the surrounding rock conditions, blasting equipment, blasting parameters, charging structure, and other conditions. Therefore, overcoming the challenge of how to adjust blasting parameters is very important for the whole tunnel construction process. The TBM method is a continuous and parallel construction method that uses integrated assembly line construction equipment to carry out a series of processes including tunneling, support, and slag discharge. Therefore, it has the advantage of fast speed and can carry out long-term deep-buried tunnel construction in the terrain environment where the drilling and blasting method cannot be used for construction [5].

With the continuous development of modern computer technology, the construction technology of engineering projects is also improving. The new computer technology is applied to the drilling and blasting construction of expressway tunnel faults. First, the geological environment is analyzed. Second, the role of drilling and blasting method and the TBM method in construction is analyzed. Furthermore, the changes in the surrounding rock of the tunnel fault during construction are analyzed. Then, the minimum smooth blasting process parameters are explored. Finally, the blasting effect data are collected at the construction site and analyzed by means of applied mechanics and numerical simulation and the optimal algorithm model of tunnel fault drilling and blasting construction is constructed. The innovation lies in the proposed expressway tunnel fault drilling and blasting construction parameter optimization model based on the combination of the Support Vector Regression (SVR) algorithm and genetic algorithm (GA). Optimization is implemented for blasting. It is proved that the proposed construction parameter optimization model not only has a short computation time and low computation cost but also has a strong blasting location optimization ability, which is very suitable for tunnel engineering, and provides a new perspective for the development of tunneling technology for road construction in the future.

## 2. Establishment of the Optimization Model of Construction Parameters

### 2.1. Analysis of Construction Geography and Landform

A tunnel is a kind of engineering building buried in the ground, which is one of the forms of using underground space. A long tunnel (a tunnel with a length of over 1 km) is selected for construction analysis. The tunnel type is an arc-shaped super long tunnel with left and right separation, which is located in Huangshan City, Anhui Province, China, and belongs to the subtropical region. The climate is a humid monsoon climate, which is characterized by a mild and humid climate, a rainy and humid climate, distinct seasonal boundaries, more precipitation, and a plum rain season [6].

The article "Stability Analysis and Construction Parameter Optimization of Tunnels in the Fractured Zone of Faults" was retracted in 2023. Reasons: signs of a paper mill; suspected computer-generated content; unreliable results or conclusions; concerns about the data.

The mountain rocks at the construction site are mainly melilite, fine sandstone, carbonaceous shale, siliceous, carbonaceous mudstone, limestone, early Yanshanian granodiorite, gabbro, and augite peridotite [7]. The main stratigraphic types are shown in Table 1.

### 2.2. Drilling and Blasting and TBM

The drilling and blasting method, as the traditional method of tunnel project construction in China, is composed of seven working procedures including measurement and positioning, perforation, charging, network login, blasting and smoke exhaust, slag removal, and tunnel support (Figure 1). The most important requirement of drilling and blasting construction is minimizing the influence of surrounding rock during blasting and the damage caused by blasting to surrounding rocks [3, 8].

It has the following advantages. A. The drilling and blasting method is flexible in construction and the construction path can be changed at any time. B. The construction scope is wide and can be used in most mountain tunnel construction projects. C. There is little investment in fixed assets in the early stage and the preparation period required by the project is very small. D. The management of the construction team is similar to that of a traditional site and no special control is required. E. There is no overlapping time for each construction process, but the process is connected quickly. F. Each process shall be carried out by its professional team. However, it also has the following disadvantages. A. The level of coordination between each type of work and each process is in great demand. B. Tunnel blasting construction will have an impact on the quality of the surrounding rock, which damages the rock and reduces its mechanical properties. Moreover, the damage generated in the later stage will develop into a damage zone, thus increasing the internal stress of rock mass and reducing the bearing capacity of the surrounding rock. C. Late support depends on the effect of blasting on construction. D. Due to its own operating characteristics, the tunnel will be overdug, which will affect the quality, efficiency, and safety of tunnel construction. E. Over excavation will increase the project cost, increase the hidden danger of operation, affect the laying of the tunnel waterproof layer, affect the operation schedule, and affect the quality of surrounding rocks. Therefore, the setting of tunnel blasting parameters is particularly important for the quality of the whole project.

The article "Stability Analysis and Construction Parameter Optimization of Tunnels in the Fractured Zone of Faults" was retracted in 2023. Reasons: signs of a paper mill; suspected computer-generated content; unreliable results or conclusions; concerns about the data.

TBM is mainly used for tunnel construction of railways, highways, water conservancy, hydropower, and so on. For hard rocks, TBM is divided into two types: open type and shield machine. It integrates tunnel excavation, support, dredging, and other construction processes to work parallelly and continuously. It is a highly integrated pipeline tunnel construction facility. This method has the advantages of fast excavation speed, short construction period, green safety, good comprehensive performance, and less supporting work and is suitable for operation in a complex geological environment. The disadvantage is that it can only be used in long tunnel operations, which requires a high management level, high preinvestment cost, high maintenance demand during operation, and high engineering cost [5].  Figure 2 shows the shield mechanism type and working procedure diagram.

### 2.3. Applied Mechanical Analysis

#### 2.3.1. Stress Calculation of Tunnel over and under Excavation

Tunnel over excavation refers to the excavation contour line on the drawing design being taken as the standard when tunneling, and the multiexcavation part that exceeds the excavation reference line is called the over excavation. The undercut part that does not reach the excavation reference line is called the undercut. As the surrounding rock in the tunnel fault is a homogeneous hard rock, the tunnel is deeply buried in the soil and the tunnel is a long tunnel. For the water purification field at initial stress, the cross-section of the tunnel is approximately circular, and its cross-section shape and coordinate system are established as shown in Figure 3.

The calculation equation of stress state *σ*_*P*_ on 0–1 axis and 0–2 axis of vertex symmetry of the contour attapulgite line is shown in equations (1) and (2), respectively. The values of radial stress and shear stress are both zero at the overcut and undercut vertex, and the calculation equation of tangential stress *σ*_*θ*_ is shown in equations (3) and (4), respectively. Equation (5) is the calculation of tangential stress *σ*_*θ*_ in other positions, and equation (6) is the calculation of circular tunnel stress in an ideal smooth model.

(1) $$\begin{array}{c} \frac{\sigma_{\theta }}{\sigma_{P}}=\frac{\gamma H}{\left(\rho^{n+1}+mC_{2}\right)/\left(\rho^{n+1}-mC_{2}\right)}\pm \left[\rho^{2m}\left(1+mC_{2}^{2}\right)\right]-m\left(n+1\right)\frac{C_{2}\rho^{n+1}\left(\rho^{n+1}+C_{2}\right)}{{\left(\rho^{n+1}-mC_{2}\right)}^{3}}, \end{array}$$

(2) $$\begin{array}{c} \frac{\sigma_{\theta }}{\sigma_{P}}=\frac{\gamma H}{\left(\rho^{n+1}+mC_{2}\right)}\pm \left[\rho^{2m}\left(1+mC_{2}^{2}\right)\left(\rho^{n+1}-mC_{2}\right)\right]-m\left(n+1\right)\frac{C_{2}\rho^{n+1}\left(\rho^{n+1}+C_{2}\right)}{{\left(\rho^{n+1}-mC_{2}\right)}^{3}}, \end{array}$$

(3) $$\begin{array}{c} \sigma_{\theta }=2\gamma H\frac{\left(1+mC_{2}\right)}{\left(1-mC_{2}\right)}, \end{array}$$

(4) $$\begin{array}{c} \sigma_{\theta }=2\gamma H\frac{\left(1-mC_{2}\right)}{\left(1+mC_{2}\right)}, \end{array}$$

(5) $$\begin{array}{c} \sigma_{\theta }=2\gamma H\frac{\left(1-m^{2}C_{2}^{2}\right)}{\left[1+m^{2}C_{2}^{2}-2mC_{2}\cos\left(m+1\right)\theta \right]}, \end{array}$$

(6) $$\begin{array}{c} \frac{\sigma_{\theta }}{\sigma_{r}}=\gamma H\left(1\pm \frac{1}{r^{2}}\right), \end{array}$$

where *γ* is the bulk density of rock mass covered by the tunnel, *H* represents the buried depth of the tunnel, *m* represents the number of overdug parameters, *C*_2_ represents the parameter of over-dug degree, *ρ* represents the characteristic coordinates of the tunnel design baseline, and *r* is the radius of the ideal circular contour. When the tangential stress *σ*_*θ*_ of 0–1 axis exceeds 2*γH*, its maximum value appears at the overcut vertex. When the tangential stress *σ*_*θ*_ of 0–2 axis does not exceed 2*γH*, its minimum value appears at the undercut vertex. Hence, over excavation will lead to a concentration of additional stress, but under excavation will not produce overstress [9].

The article "Stability Analysis and Construction Parameter Optimization of Tunnels in the Fractured Zone of Faults" was retracted in 2023. Reasons: signs of a paper mill; suspected computer-generated content; unreliable results or conclusions; concerns about the data.

#### 2.3.2. Mechanical Standard of Tunnel over and under Excavation

In the tunnel excavation of hard rock mass, the overdigging height should be less than 0.02–0.25 m. On this basis, it is guaranteed that the attached stress concentration will not affect or have little effect on the stability of the surrounding rock, which basically meets the national and industry standards in the tunnel design and construction code. The calculation between the overbreak standard deviation and the allowable overbreak height is shown in equations (7) and (8).

(7) $$\begin{array}{c} h=4{\left(D_{a}R\right)}^{0.5}, \end{array}$$

(8) $$\begin{array}{c} s^{2}=\frac{\sum_{i=1}^{n}\left(x_{i}-\bar{x}\right)}{n-1}, \end{array}$$

where *D*_*a*_ is the variance of the tunnel overcut value, *R* is the equivalent radius of the tunnel, *x*_*i*_ is the *x*-th sample value, and $\bar{x}$ is the average value of *x*_*i*_.

Equation (9) is the shear resistance calculation of surrounding rock at any section, and equation (10) is the shear resistance of an idealized uniform rod.

(9) $$\begin{array}{c} T=\sigma_{n}f_{r}\frac{ab-A_{s}}{\sin\;\theta }+c_{r}\frac{ab-A_{s}}{\sin\;\theta }+\tau_{s}\frac{A_{s}}{\sin\;\theta }, \end{array}$$

(10) $$\begin{array}{c} T=\sigma_{n}f_{r}\frac{ab}{\sin\;\theta }+c\frac{ab}{\sin\;\theta }, \end{array}$$

where *f* is the friction coefficient of the shelter, *c* is the cohesion of the rock mass, *τ*_*s*_ is the shear strength, *A*_*s*_ represents the cross-sectional area, *ab* represents the average distance of the rod, and *θ* represents the included angle between the cross-section and the rod. The calculation of the unidirectional compressive strength of the member is shown in equation (11), and the equivalent deformation modulus and shear modulus of the surrounding rock are shown in equations (12) and (13).

(11) $$\begin{array}{c} c=c_{r}+\tau_{s}\frac{A_{s}}{ab}, \end{array}$$

(12) $$\begin{array}{c} \tau_{s}=\frac{\sigma_{s}\pi d^{2}}{4\sqrt{3}}, \end{array}$$

(13) $$\begin{array}{c} \sigma_{c}=\frac{2\;\cos\;\phi }{1-\sin\;\phi }, \end{array}$$

where *τ*_*s*_ is the yield strength of the rod, *d* is the diameter of the rod, and *f* and *c* represent the equivalent friction coefficient and equivalent cohesion, respectively.

The article "Stability Analysis and Construction Parameter Optimization of Tunnels in the Fractured Zone of Faults" was retracted in 2023. Reasons: signs of a paper mill; suspected computer-generated content; unreliable results or conclusions; concerns about the data.

#### 2.3.3. Numerical Simulation

The explosion is an energy conversion process that converts chemical energy into kinetic energy. It refers to a very short process in which a small amount of solid or liquid reacts in a confined space to generate a large amount of gas, which rapidly increases the volume of reaction products and generates shock waves and extremely high heat. High-density energy explosives are not only widely used in the military industry but also in daily life. The destructive nature of the explosion makes the cost of the experiment too high and the test process is also very complex. Due to the limited measurement methods and observation conditions, civil explosion research is limited. In addition, in experiments and observations, there will be many unpredictable interference conditions, so the repeatability is not good. All kinds of situations will affect the in-depth and meticulous development of testing work. With the rapid development of computer manufacturing technology and information technology, numerical simulation of explosive mechanics has developed by leaps and bounds. At the same time, mathematical models for calculating explosions have become more sophisticated and accurate. The numerical simulation process is gradually rationalized and its advantages are gradually revealed. Numerical simulation can arbitrarily change the conditions and parameters of numerical simulation, combined. After the combination with the mathematical analysis method, some of the most important parameter variation trends can be found, thus providing powerful help for experimental research, reducing the number of experiments. Compared with experiments, its cost is lower and it is not affected and restricted by natural conditions [10, 11].

The article "Stability Analysis and Construction Parameter Optimization of Tunnels in the Fractured Zone of Faults" was retracted in 2023. Reasons: signs of a paper mill; suspected computer-generated content; unreliable results or conclusions; concerns about the data.

In this experiment, the dynamic finite element method is used to solve mathematical equations, and the ANSYS/LS-DYNA dynamic finite element program is used, which is very suitable for solving the impact dynamics problems of nonlinear structures such as an explosion. The Lagrange shared node algorithm is chosen for simulation and analysis.  Figure 4 shows the finite element equation solving process and hourglass control.

### 2.4. Intelligent Optimization Model of Drilling and Blasting Construction Parameters

SVR algorithm combined with GA is used to construct the model.

#### 2.4.1. SVR Algorithm

SVR is an important application branch of support vector machines. The SVR regression refers to finding a regression plane so that all the data points in a set are closest to the plane. It is a linear regression algorithm. The linear regression refers to fitting samples with linear functions in a vector space. In this model, the synthetic distance between the actual position of all samples and the linear function is taken as the loss, and the parameters of the linear function are obtained by minimizing the loss. For linear regression, if the sample does not fall within the specified range of the model, the loss will be calculated. SVR creates a “spacing band” on both sides of the linear function. The spacing is also known as tolerance deviation, which is a manually set empirical value, and the loss is not calculated for all samples falling into the spacing band.

For all samples falling into the interval band, the loss is not calculated. Only those outside the interval band are included in the loss function. Then, the model is optimized by minimizing the width and total loss of the spacer band. Only those red samples (either outside or on the edge of the isolation zone) are counted as final losses [12–14].  Figure 5 shows the SVR schematic and functional representation.

Figure 5 shows the basics of the SVR. The model function *f*(*x*)=*ωx*+*b* is the requested one. *ωx*+*b*+*ε* and *ωx*+*b* − *ε* are the upper and lower edges of the separation zone, respectively. *ξ*^*∗*^ is the difference between the projection from the sample point below the lower edge of the isolation belt to the lower edge of the isolation belt and the *y* of the sample point, *ω*, *b* is the setting parameter, and *x* is the independent variable of the sample.

The article "Stability Analysis and Construction Parameter Optimization of Tunnels in the Fractured Zone of Faults" was retracted in 2023. Reasons: signs of a paper mill; suspected computer-generated content; unreliable results or conclusions; concerns about the data.

Equations (14) and (15) show the corresponding calculations.

(14) $$\begin{array}{c} \xi_{i}=y_{i}-\left(f\left(x_{i}\right)+\varepsilon \right),\;\text{if}\left\{y_{i}>f\left(x_{i}\right)+\varepsilon \right\}\\ \xi_{i}=0,\;\left\{\text{otherwise}\right\}, \end{array}$$

(15) $$\begin{array}{c} \xi_{i}{}^{*}=\left(f\left(x_{i}\right)-\varepsilon \right)-y_{i},\;\text{if}\left\{y_{i}<f\left(x_{i}\right)-\varepsilon \right\}\\ \xi_{i}{}^{*}=0,\;\left\{\text{otherwise}\right\}, \end{array}$$

For any sample, *x*_*i*_, if it is in the isolation band or on the edge of the isolation band, then *ξ*_*i*_^*∗*^ and *ξ*_*i*_ are 0. If it is above the upper edge of the isolation band, then *ξ*_*i*_ > 0, *ξ*_*i*_^*∗*^=0. If it is below the lower edge of the quarantine zone, then *ξ*_*i*_=0, *ξ*_*i*_^*∗*^=0.

Thus, for the quadratic optimization problem of construction, the Lagrange function is used in equation (16). Equation (17) is the solution condition, and the maximization function is shown in equation (18).

(16) $$\begin{array}{c} L\left(w,b,\xi ,\xi^{*},\alpha ,\alpha^{*},\gamma ,\gamma^{*}\right)=\frac{1}{2}w^{*}w+C\sum_{i=1}^{k}\left(\xi_{i}+\xi_{i}^{*}\right)\\ -\sum_{i=1}^{k}\alpha_{i}\left[\xi_{i}+\varepsilon -y_{i}+f\left(x_{i}\right)\right]-\sum_{i=1}^{k}\left(\xi_{i}\gamma_{i}+\xi_{i}{}^{*}\gamma_{i}{}^{*}\right), \end{array}$$

(17) $$\begin{array}{c} \sum_{i=1}^{k}\left(\alpha_{i}-\alpha_{i}^{*}\right)=0,\\ w=\sum_{i=1}^{k}\left(\alpha_{i}-\alpha_{i}^{*}\right)x_{i},\\ C-\alpha_{i}-\gamma_{i}=0,\\ C-\alpha_{i}^{*}-\gamma_{i}^{*}=0, \end{array}$$

(18) $$\begin{array}{c} W\left(\alpha ,\alpha^{*}\right)=-\frac{1}{2}\sum_{i,j=1}^{k}\left(\alpha_{i}-\alpha_{i}^{*}\right)\left(\alpha_{j}-\alpha_{i}^{*}\right)\left(x_{i}*x_{j}\right)+\sum_{i=1}^{k}\left(\alpha_{j}-\alpha_{i}^{*}\right)y_{i}-\sum_{i=1}^{k}\left(\alpha_{j}+\alpha_{i}^{*}\right)\varepsilon . \end{array}$$

where *ω*, *b*, *α*, *ε*, *γ* are parameters.

#### 2.4.2. GA

GA is a computational model that simulates the biological evolution process of natural selection and the genetic mechanism of Darwin's biological evolution. It is a method to search for the optimal solution by simulating the natural evolution process. It originated from the computer simulation of biological systems; it is a stochastic global search optimization method. It stimulates the phenomena of replication, crossover, and mutation that occur in natural selection and heredity, starting from any initial population and producing a group of individuals better suited to the environment through random selection, crossover, and mutation. In this way, the population evolves to better and better areas of the search space, so that the evolution of continuous reproduction, and finally, converges on a group of individuals who are the most adaptable to the environment, so as to find a good solution to the problem.

The article "Stability Analysis and Construction Parameter Optimization of Tunnels in the Fractured Zone of Faults" was retracted in 2023. Reasons: signs of a paper mill; suspected computer-generated content; unreliable results or conclusions; concerns about the data.

GA takes all individuals in a population as subjects and uses a randomization technique to guide a coded parameter space to search efficiently. Selection, crossover, and variation constitute the genetic operations of a genetic algorithm. The core content of a genetic algorithm is composed of five elements, namely, parameter coding, initial population setting, fitness function design, genetic operation design, and control parameter setting [15, 16]. The algorithm flowchart is shown in Figure 6.

The objective function of the GA is shown in equation (19), and the fitness function is shown in equation (20).

(19) $$\begin{array}{c} s^{2}=\frac{1}{n}\sum_{i=1}^{n}{\left(f\left(x_{i}\right)-y_{i}\right)}^{2}, \end{array}$$

(20) $$\begin{array}{c} g\left(x\right)=\exp\left\{-0.05\max\left[\frac{\left|f\left(x_{i}\right)-y_{i}\right|}{y_{i}}\right]\right\}, \end{array}$$

where *f*(*x*_*i*_) is the SVR output value of the *i*-th test sample during training, *y*_*i*_ is the sample value, and *n* represents the number of test samples.

#### 2.4.3. Evolutionary Support Vector Machine Algorithm

GA is combined with the SVR algorithm and its algorithm steps are shown in Figure 7.

### 2.5. The Simulation

The ANSYS/LS-DYNA dynamic finite element program is utilized, and a model is established to simulate the smooth blasting experiment on the tunnel face. The influence data of blasting on surrounding rock are obtained, and the experimental results of photo-explosion are finally obtained to put forward the optimization parameter model. Two three-dimensional solid element types are established in ANSYS/LS-DYNA. If the 8-node Solid 164 and the 10-node Solid 168 are used to divide the element types, irregular 4-hedral network nodes cannot be obtained. Therefore, Solid 168 is used as the cell type to divide the mesh and the regular surface mesh is obtained.

## 3. Test of Construction Parameter Optimization Model

### 3.1. Experimental Results of Light Explosion

In Figure 8, ten representative section points are randomly selected to verify the optical explosion experimental results.

Figure 8(a) shows the average distance between peripheral eyes, the average of auxiliary eyes, and the average row distance, and Figure 8(b) shows the horizontal convergence, arch subsidence, arch foot loosening, and arch waist loosening. Therefore, the ten points selected are relatively representative and their average value is relatively representative. The average distance between peripheral eyes was 50 cm, and the average distance between auxiliary eyes was 85 cm. The average row spacing is about 60 cm, but the distribution of horizontal convergence and vault subsidence is relatively scattered. The distribution of arch foot looseness and arch waist looseness is about 1.4 m, but the distribution is still relatively scattered. The above data set is used as the data set of the drilling and blasting construction parameter optimization model.

The article "Stability Analysis and Construction Parameter Optimization of Tunnels in the Fractured Zone of Faults" was retracted in 2023. Reasons: signs of a paper mill; suspected computer-generated content; unreliable results or conclusions; concerns about the data.

### 3.2. Establishment of the Intelligent Model of a Borehole Position

Figure 9 shows the weight of optical explosion investigation index, and Figure 10 shows the optimal drilling and blasting process parameters.

In Figure 9, the weight of the light explosion index is 0.2 for horizontal convergence, 0.4 for arch subsidence, 0.15 for arch foot loosening, and 0.25 for arch waist loosening. The population size of GA is 20, and the optimal SVR model parameters are obtained after 400 generations of evolution, with C being 831.9, the slope parameter 41.03, the outcome parameter 0.8902, and fitness 0.907. Therefore, the mean distance between peripheral eyes is 66–67 cm, the mean distance between auxiliary eyes is 60–75 cm, and the mean distance between row eyes is 64–71 cm. The fitness of both eyes is 1.

## 4. Conclusion

This paper optimizes the drilling and blasting construction method under the background of modern computer technology. First, this paper analyzes the construction geology and landforms. Second, the advantages and disadvantages of the drilling and blasting method and TBM construction are compared, and their adaptability in the current construction environment is analyzed. In addition, the influence of drilling and blasting methods on surrounding rocks and excavation conditions is analyzed by mechanics. Then, this paper discusses the minimum smooth blasting process parameters under these conditions, combines the SVR algorithm with the genetic algorithm, constructs an evolutionary support vector machine algorithm for parameter optimization, and constructs the tunnel faults drilling and blasting process parameter optimization algorithm model. Finally, this paper also takes the collected optical explosion experimental data as the training data set, trains the construction model, and obtains the best parameters required for drilling and blasting construction.

Although this experiment has basically achieved the expected research objectives and achieved some valuable research conclusions, there are still many deficiencies in the research work and the conclusions are limited by the following two factors. The sites of different rock masses are insufficient. The long-term construction data have not been collected, which also points out the direction for our future research. In the future, we will focus on two aspects. We will collect and simulate data of different rock masses. We will expand the size of the data set to increase the number of training sessions and improve it through better algorithm prediction.

The article "Stability Analysis and Construction Parameter Optimization of Tunnels in the Fractured Zone of Faults" was retracted in 2023. Reasons: signs of a paper mill; suspected computer-generated content; unreliable results or conclusions; concerns about the data.

## Figures and Tables

**Figure 1:** The whole process.

**Figure 2:** Shield mechanism type and working procedure diagram. (a) Shield machine structure diagram. (b) Shield machine working procedure diagram.

**Figure 3:** Contour of excavation.

**Figure 4:** Numerical simulation process. (a) Finite element equation solving process and (b) model hourglass control.

**Figure 5:** SVR algorithm schematic diagram. (a) SVR schematic diagram and (b) function expression diagram.

**Figure 6:** Algorithm flowchart.

**Figure 7:** Algorithm steps.

**Figure 8:** Verification of optical explosion experimental results. (a) Eye spacing and (b) variation value.

**Figure 9:** Weight of the optical explosion inspection index.

**Figure 10:** Optimal drilling and blasting process parameters.

**Table 1:** Stratigraphic rock types.

Type	Composed kinds	Component name	Rock property	Thickness
A	2	Hypomere	Gray black light metamorphic siltstone and lithic feldspar quartz sandstone interbedded with the homochromatic silty slate and sandy phyllite	932.0 m
		Epimere	Gray and gray-green millennium-like siltstone intercalated with the same color sand-bearing millenniolite and silty millenniolite	968.0 m

B	3	Lower part	Gray purplish red conglomerate, gravel feldspar quartz sandstone, fine sandstone, and siltstone	576.9 m

C	1	All part	Crushed silty clay	0.3–3.0 m

D	1	Early Yanshanian invasion	Biotite granodiorite, gneiss structure, and massive structure	32 km

## Data Availability

The data used to support the findings of this study are available from the corresponding author upon request.
